# High-Sensitivity C-Reactive Protein and Ischemic Stroke in Patients with Nonalcoholic Fatty Liver Disease: A Prospective Study

**DOI:** 10.1155/2022/9711712

**Published:** 2022-03-30

**Authors:** Meng Jia, Yingxin Shi, Yuemeng Wang, Mei Wang, Liang Zhang, Qingjuan He, Tao Yuan

**Affiliations:** ^1^Department of Geriatrics, Qingdao Eighth People's Hospital, Qingdao, Shandong 266121, China; ^2^Intensive Care Unit, Qingdao Eighth People's Hospital, Qingdao, Shandong 266121, China; ^3^Department of Gastroenterology, Qingdao Eighth People's Hospital, Qingdao, Shandong 266121, China

## Abstract

**Background and Aims:**

Inflammation is involved in the pathophysiology of ischemic stroke. The aim of this prospective study was to evaluate the association of hs-CRP with incident ischemic stroke in patients with nonalcoholic fatty liver disease (NAFLD).

**Methods:**

A sample of 318 participants without previous strokes was included in this study. Hs-CRP levels and other potential confounding factors were measured at baseline. NAFLD was performed by abdominal ultrasound after excluding secondary causes for fat accumulation. According to baseline hs-CRP concentrations, participants were categorized into 3 groups: level 1 (<1.0 mg/L), level 2 (1.0 to <3.0 mg/L), and level 3 (≥3.0 mg/L). The outcome of interest was the first occurrence of an ischemic stroke. Cox proportional hazards models were used to analyze hazard ratios (HRs) and 95% confidence intervals (CIs) of incident ischemic stroke, after adjusting for potential confounders.

**Results:**

The mean age of 318 participants with NAFLD was 71.1 ± 6.7 years, and 55.3% of them were male. Among 318 individuals with NAFLD, 115 (36.2%) of them had an hs-CRP value <1 mg/L (level 1), 105 (33.0%) had an hs-CRP value between 1 and 3 mg/L (level 2), and 98 (30.8%) belonged to level 3 (hs-CRP ≥3 mg/L). Over a median of 5.60 years of follow-up, 47 incident ischemic stroke events were documented in 318 patients with NAFLD. After full adjustment for confounding factors, compared with participants in the level 1 group (hs-CRP<1.0 mg/L), the HRs of those in the level 2 group (1.0 to <3.0 mg/L) and the level 3 group (≥3.0 mg/L) were 1.77 (95% CI: 0.94–2.98) and 2.45 (95% CI: 1.37–5.77) for developing ischemic stroke, respectively.

**Conclusions:**

Elevated hs-CRP levels were associated with an increased risk of ischemic stroke among patients with NAFLD.

## 1. Introduction

Ischemic stroke approximately accounts for 70–80% of strokes, which is the second most common cause of death and the third most common cause of disability in the world [1]. In 2013, there were almost 18.3 million patients with previous ischemic stroke, 3.3 million deaths from ischemic stroke, and 6.9 million new ischemic strokes worldwide [2]. An international study of stroke costs shows that the estimated expenditure for stroke was about 3% of total health care expenditures, which is similar among eight developed countries [3]. Thus, the need to take more efficient stroke prevention and treatment strategies is urgent. Nonalcoholic fatty liver disease (NAFLD), a common cause of liver disease, could be an independent risk factor for future ischemic stroke [4]. The prevalence of NAFLD is 25.24% globally, with many metabolic comorbidities including obesity (51.34%), type 2 diabetes (22.51%), dyslipidemia, and metabolic syndrome [5]. A recent meta-analysis with 34,043 adult individuals demonstrated that patients with NAFLD were more likely to have incident fatal and nonfatal cardiovascular disease events [6]. Furthermore, a better understanding of the potential mechanism between NAFLD and ischemic stroke might have important clinical implications for future healthcare policies.

Inflammation response is likely to play an essential role in the pathogenesis and progression of ischemic stroke [7]. C-reactive protein (CRP) using a high-sensitivity assay (high-sensitivity CRP, hs-CRP), a low-grade chronic inflammation biomarker, has been demonstrated to be associated with an increased risk of ischemic stroke [8]. CRP, an acute-phase reactive protein, is a blood constituent of the pentraxin family and is synthesized by the liver [9]. CRP is thought to be involved in activating platelets and complement proteins by interacting with other mediators [10, 11]. A meta-analysis of 54 long-term prospective studies indicated that the risk ratio (RR) of per standard deviation higher log(*e*) CRP was 1.27 (1.15–1.40) for ischemic stroke after adjusting for conventional risk factors [12]. A case-control study of 472 strokes showed that the adjusted odds ratio (OR) of the last third of CRP level was 1.39 (95% CI: 1.05–1.85) for recurrent ischemic stroke [13]. By contrast, the Northern Manhattan Study (NOMAS) of 2,240 stroke-free community participants suggested that hs-CRP could predict mortality but not ischemic stroke [14]. Consequently, the controversial evidence of hs-CRP in ischemic stroke makes the role of hs-CRP levels in the clinical setting remain unclear.

The objective of this study is to examine the association of hs-CRP levels with the occurrence of ischemic stroke among patients with nonalcoholic fatty liver disease, after adjusting for potential confounding factors.

## 2. Methods

### 2.1. Study Population

The current study was a hospital-based prospective cohort study aiming to investigate the relationship between NAFLD and ischemic stroke. From April 2009 to June 2011, participants aged ≥18 years were recruited from the outpatient department in our hospital. After excluding patients with acute infection, unknown fever, cancer, autoimmune diseases, severe kidney and liver dysfunction, hypercoagulable state, or hematological diseases, 658 patients were eligible for the study. Each participant was scheduled to undergo a baseline survey, including questionnaire evaluation, physical examinations, biochemical tests, and abdominal ultrasound. The details of 318 patients with NAFLD enrolled in the analysis are shown in Figure 1.

All participants have signed informed consent. This study protocol was approved by the ethics committee of local hospital.

### 2.2. Baseline Data Collection

Participants' information was obtained by using standard questionnaires, including age, sex, smoking status, alcohol consumption, and disease history (such as hypertension, diabetes, and dyslipidemia). Each participant underwent a physical examination of height and weight, and BMI was calculated by body weight (kg) divided by height square (m^2^). After participants were seated silently for 15 minutes, systolic blood pressure (SBP) and diastolic blood pressure (DBP) were measured by using an automatic blood pressure meter. Venous blood samples were drawn in the morning after an 8-hour overnight fast. Blood levels of alanine transferase (ALT), aspartate transferase (AST), total cholesterol (TC), triglyceride (TG), low-density lipoprotein cholesterol (LDL-C), high-density lipoprotein cholesterol (HDL-C), creatinine, and uric acid (UA) were measured by using an AutoAnalyzer (Hitachi 747; Japan) at the clinical laboratory of a local hospital. The concentration of hs-CRP was assessed by high-sensitivity nephelometry assay (Cias Latex CRP-H; Japan). The lower limit of detection was 0.10 mg/L. The intraassay coefficient of variation was 6.5%, and the interassay coefficient of variation was 4.8%.

### 2.3. Assessment of NAFLD

NAFLD was defined as hepatic steatosis assessed by abdominal ultrasound without causes for secondary fat accumulation. Abdominal ultrasound was performed by well-trained radiologists who were blinded to clinical characteristics and laboratory tests. Excessive alcohol intake was determined as >210 g/week in men and >140 g/week in women based on the guideline recommendation [15].

### 2.4. Follow-Up and Ischemic Stroke Ascertainment

From the baseline survey, the follow-up of study participants was continued until the incidence of stroke, or June 30, 2019, whichever came first. We contacted study participants or their authorized persons by interview or telephone every year. The outcome of interest was the first occurrence of an ischemic stroke. The ascertainment of ischemic stroke was determined by an experienced clinician after a systematic review of clinical symptoms, physical signs, and brain computed tomography scans or magnetic resonance imaging.

### 2.5. Statistical Analysis

All patients were categorized into three groups according to hs-CRP concentrations: level 1 (<1.0 mg/L), level 2 (1.0-<3.0 mg/L), and level 3 (≥3.0 mg/L) [8]. Categorical variables were described by frequencies and percentages, and compared using chi-squared tests. Continuous variables with a skewed distribution were expressed as median (25% and 75%) and compared using the Kruskal–Wallis test. Continuous variables with normal distributions were presented as mean ± standard deviation (SD) and compared using the student's *t*-test or the 1-way ANOVA test. Kaplan–Meier curves were used to present the time to incident ischemic stroke event for each hs-CRP group. We used Cox proportional hazards models to estimate the independent association of hs-CRP levels with the occurrence of ischemic stroke, after adjusting for potential confounding factors in three models, respectively. The potential confounding factors included age, gender, BMI, history of hypertension, diabetes, dyslipidemia, SBP, DBP, TC, TG, LDL-C, ALT, AST, creatinine, and UA. A significant level was set as *P* < 0.05 (2-sided). Statistical analyses were performed with IBM SPSS Statistics 21.0.

## 3. Results

658 patients were enrolled in the study, but only 619 patients completed the baseline examination (Figure 1). We excluded 147 subjects without abdominal ultrasound data (*n* = 102) and hs-CRP values (*n* = 45), 27 patients with previous ischemic stroke, 112 patients with excessive alcohol consumption, and 15 patients who lost follow-up. Finally, a total of 318 patients with nonalcoholic fatty liver disease were included in the study (Figure 1).

The mean age of 318 participants with NAFLD was 71.1 ± 6.7 years, and 55.3% of them were male. Baseline characteristics of the study participants based on the hs-CRP levels are shown in Table 1. Among 318 individuals with NAFLD, 115 (36.2%) of them had an hs-CRP value <1 mg/L (level 1), 105 (33.0%) had an hs-CRP value between 1 and 3 mg/L (level 2), and 98 (30.8%) belonged to level 3 (hs-CRP ≥3 mg/L). Compared with patients in level 1, patients in level 3 were more likely to be older, have a higher BMI, and have a history of hypertension and dyslipidemia. Individuals with hs-CRP ≥3 mg/L had a higher level of blood pressure, TC, LDL-C, and serum UA than individuals with hs-CRP <1 mg/L. However, there was no significant difference among participants in three hs-CRP subgroups in the proportion of gender, diagnosed diabetes, and the concentration of TG, HDL-C, ALT, AST, and creatinine.

Table 2 shows the hs-CRP levels in different subgroups. Participants aged ≥75 years had higher hs-CRP levels of 2.37 (1.01, 3.73) than participants aged <65 years. Besides, subjects with a BMI ≥28 kg/m^2^ had higher hs-CRP levels of 2.79 (2.07, 4.51) than subjects with a BMI <24 kg/m^2^. The levels of hs-CRP were not significantly associated with hypertension. However, the levels of hs-CRP were higher with prevalent diabetes and dyslipidemia.

After a median follow-up of 5.60 years, we identified 47 incident ischemic stroke events among 318 patients with nonalcoholic fatty liver disease. The Kaplan–Meier curve revealed that NAFLD patients with higher hs-CRP levels appeared to separate from the other groups throughout the follow-up period (Figure 2). The Logrank and Breslow tests suggested that the survival distributions of these three groups differed significantly (Logrank test *P*=0.006; Breslow test *P* < 0.001), indicating that the mean time for incident ischemic stroke event in NAFLD patients with hs-CRP concentration ≥3 mg/L was significantly shorter compared to NAFLD patients with hs-CRP concentration <3 mg/L (Figure 2).

In a Cox proportional hazards analysis with patients in level 1 as the reference group, the patients with hs-CRP in level 3 were independently associated with the high risk of ischemic stroke (Table 3). Compared to participants with hs-CRP <1 mg/L (level 1), the adjusted HRs for the risk of ischemic stroke was 2.07 (95% CI: 0.90–4.72) in the level 2 group and 3.30 (95% CI: 1.52–7.14) in the level 3 group, after adjusting age and gender in model 1 (P for trend = 0.006). Model 2 adjusted for model 1 and for BMI, history of hypertension, diabetes, and dyslipidemia. After adjusting for a series of potential confounding factors in model 3, the adjusted HR for patients with hs-CRP of 1 to <3 mg/L was 1.77 (95%CI, 0.94–2.98), and the adjusted HR for patients with hs-CRP >3 mg/L was 2.45 (95%CI, 1.37–5.77) compared to patients with hs-CRP <1 mg/L (P for trend = 0.011).

## 4. Discussion

In this prospective study of 318 patients with NAFLD, after a median of 5.6 years of follow-up, we observed an independent association of hs-CRP level with the occurrence of ischemic stroke. High hs-CRP concentration was significantly associated with elevated risk of ischemic stroke, after adjusting a series of potential confounding factors including demographic characteristics, medical history, and metabolic parameters. Our results support the validity of circulating hs-CRP as a clinical biomarker to detect subjects at high risk of ischemic stroke who are likely to benefit from primary prevention strategies among patients with NAFLD.

The association of hs-CRP and ischemic stroke in our study was in accordance with the findings in the Cardiovascular Health Study. The Cardiovascular Health Study of 5417 individuals aged 65 years or older without previous stroke, after 10.2 years of follow-up, found that the adjusted HR in the 4th quartile of CRP level was 1.60 (95% CI: 1.23–2.08) for ischemic stroke relative to the 1st quartile [16]. In addition, an international, multicenter, prospective study indicated that, after adjusting for demographics characteristics and risk factors, patients with hs-CRP >4.86 mg/L (the top quartile) were at elevated risk of recurrent ischemic stroke (adjusted HR: 2.32; 95% CI: 1.15–4.68) [17]. Other studies relating CRP levels to ischemic stroke have shown contrary results. The Northern Manhattan Study (NOMAS) showed that, compared with community participants with hs-CRP <1 mg/L, the adjusted HR of those with hs-CRP >3 mg/L was 1.20 (95% CI: 0.78–1.86) for an elevated risk of ischemic stroke [14]. Moreover, a previous study of 467 patients with first ischemic stroke revealed that hs-CRP level was not associated with the occurrence of recurrent stroke after adjusting for confounders [18]. The variation between these earlier studies is likely attributed to differences in sample size, different cutoff points of hs-CRP, selection of study populations, and the prevalence of comorbid conditions.

This observational study could not address the potential mechanisms of hs-CRP in ischemic stroke, but there are several studies supporting an underlying link between hs-CRP and ischemic stroke. CRP might be involved in the pathogenesis of chronic ischemia by quenching the production of nitric oxide (NO) and inhibiting angiogenesis [19]. Besides, CRP has been documented to play an important role in atherogenesis by elevating the levels of endothelin-1, cell adhesion molecules, and interleukin-8 in endothelial cells and inducing tissue factor secretion in monocyte-macrophages [20].

The association between hs-CRP and ischemic stroke was examined in an apparently healthy population [21], in participants with hypertension and diabetes [22], but not well established in patients with NAFLD. Our study in patients with NAFLD is consistent with a previous prospective study, which showed elevated gamma-glutamyltransferase (GGT) levels, mostly due to NAFLD, are associated with an increased risk of stroke independent of established cardiovascular risk factors [23]. A prospective cohort study further demonstrated that, after a median of 10.34 years of follow-up, the existence of NAFLD was associated with a higher risk of future ischemic stroke events (hazard ratio: 1.16; 95% CI: 1.08–1.50), and the severity of NAFLD was also associated with a higher risk of developing ischemic stroke [4]. However, a cross-sectional study of 1277 subjects showed that NAFLD was not associated with the prevalence of lacunar infarct in obese participants [24].

The potential mechanisms underlying the relationship of NAFLD with stroke include insulin resistance, fatty acid and lipoprotein metabolism, and endothelial dysfunction [25]. In addition, the progression of NAFLD is accompanied by activating hepatic and systemic inflammatory reactions, which are closely related to the increased risk of ischemic stroke [26]. This present study provided evidence that NAFLD might be associated with an increased risk of ischemic stroke by elevating hs-CRP levels.

The main strength of this study is the well-characterized prospective cohort of participants with a series of metabolic covariates assessed in standardized ways by well-trained healthcare providers. However, several limitations need to be acknowledged. Firstly, we did not evaluate the severity of NAFLD, which might be a risk factor for ischemic stroke. However, a previous study showed that patients with severe NAFLD had a higher concentration of hs-CRP than those with mild NAFLD, and the hs-CRP level might reflect the severity of NAFLD [4]. Therefore, we might suppose that the absence of data on the severity of NAFLD does not affect our main findings. Secondly, this analysis included a hospital-based population, so the generalizability of our results to community individuals needs to be cautious. Third, this is an observational study. We could not demonstrate the causal relationship of hs-CRP and ischemic stroke in NAFLD patients. Intervention studies with a large sample size are needed to confirm our results.

Overall, in this prospective study, elevated hs-CRP levels were associated with an increased risk of ischemic stroke among patients with NAFLD. Our findings supported that hs-CRP might be used as a potential biomarker and therapeutic target for ischemic stroke.

## Figures and Tables

**Figure 1:** Flowchart of this study.

**Figure 2:** Kaplan–Meier curves of incident ischemic stroke by different hs-CRP levels.

**Table 1:** Baseline characteristics of the study participants according to hs-CRP levels.

Variables	Baseline hs-CRP group			*P* value
	Level 1 (<1 mg/L)	Level 2 (1 to <3 mg/L)	Level 3 (≥3 mg/L)	
*n*	115	105	98	—
Age, y	69.7 ± 6.8	71.2 ± 5.9	72.1 ± 7.2	0.021
Male, *n* (%)	65 (56.5)	57 (54.3)	54 (55.1)	0.073
BMI, kg/m^2^	24.1 ± 2.7	25.4 ± 3.1	25.1 ± 3.7	0.032
Hypertension, *n* (%)	41 (35.7)	37 (35.2)	40 (40.8)	0.003
Diabetes, *n* (%)	15 (13.0)	17 (16.2)	14 (14.3)	0.104
Dyslipidemia, *n* (%)	44 (38.3)	31 (29.5)	47 (48.0)	<0.001
SBP, mmHg	132.5 ± 17.1	136.7 ± 14.2	143.1 ± 16.8	0.007
DBP, mmHg	71.3 ± 11.2	75.4 ± 10.7	78.2 ± 13.1	0.003
TC, mmol/L	4.71 ± 1.07	5.13 ± 1.45	5.92 ± 1.41	<0.001
TG, mmol/L	1.59 (0.88, 2.04	1.73 (0.75, 2.17)	1.64 (1.09, 2.21	0.129
HDL-C, mmol/L	1.02 ± 0.31	0.95 ± 0.41	0.89 ± 0.37	0.251
LDL-C, mmol/L	2.71 ± 0.55	2.99 ± 0.74	3.41 ± 0.42	<0.001
ALT, IU/L	21.3 ± 13.7	22.6 ± 11.6	24.5 ± 8.7	0.322
AST, IU/L	22.1 ± 9.2	24.1 ± 8.8	23.4 ± 7.9	0.211
Creatinine, *μ*mol/L	70.5 ± 22.1	73.4 ± 19.5	74.5 ± 20.2	0.105
UA, *μ*mol/L	321.2 ± 95.4	344.9 ± 79.4	364.4 ± 88.5	<0.001
hs-CRP, mg/L	0.68 (0.37, 0.81)	1.74 (1.21, 2.31)	4.74 (3.91, 6.22)	<0.001

BMI, body mass index; SBP, systolic blood pressure; DBP, diastolic blood pressure; TC, total cholesterol; TG, triglyceride; LDL-C, low density lipoprotein cholesterol.

**Table 2:** Comparisons of hs-CRP levels by different subgroups.

	hs-CRP, mg/L	*P* value
	Median (interquartile range)	
Age, *y*		0.032
<65	1.49 (0.74, 2.01)	
65 to <75	1.73 (0.92, 2.34)	
≥75	2.37 (1.01, 3.73)	
Gender		0.304
Male	1.82 (0.91, 2.41)	
Female	1.74 (0.89, 2.33)	
BMI, kg/m^2^		<0.001
<24	1.01 (0.41, 1.42)	
24 to <28	1.74 (0.71, 2.32)	
≥28	2.79 (2.07, 4.51)	
Hypertension		0.087
Yes	2.47 (0.91, 3.44)	
No	1.98 (1.14, 2.99)	
Diabetes		0.013
Yes	2.59 (1.08, 3.07)	
No	1.71 (0.92, 2.49)	
Dyslipidemia		<0.001
Yes	2.19 (0.94, 3.11)	
No	1.48 (0.71, 2.41)	

BMI, body mass index.

**Table 3:** Hazard ratios (HRs) for ischemic stroke by different hs-CRP levels.

	Baseline hs-CRP group			P for trend
	Level 1 (<1 mg/L)	Level 2 (1 to <3 mg/L)	Level 3 (≥3 mg/L)	
Cases, *n*	9/115	15/105	23/98	—
Incidence rate	7.83	14.29	23.47	—
Model 1, HR (95% CI)	Reference	2.07 (0.90, 4.72)	3.30 (1.52, 7.14)	0.006
Model 2, HR (95% CI)	Reference	1.98 (0.92, 3.15)	2.97 (1.43, 6.51)	0.009
Model 3, HR (95% CI)	Reference	1.77 (0.94, 2.98)	2.45 (1.37, 5.77)	0.011

Model 1: adjusted for age and gender. Model 2: adjusted for Model 1 and for BMI, history of hypertension, diabetes, and dyslipidemia. Model 3: based on model 2, further adjusted for SBP, DBP, TC, TG, LDL-C, ALT, AST, creatinine, and UA.

## Data Availability

The analysed data sets generated during the study are available from the corresponding author on reasonable request.
